# Research on Probability Distribution of Short-Term Photovoltaic Output Forecast Error Based on Numerical Characteristic Clustering

**DOI:** 10.1155/2022/5355286

**Published:** 2022-02-01

**Authors:** Peng Yan, Chenmeng Xiang, Tiecheng Li, Xuekai Hu, Wen Zhou, Lei Wang, Liang Meng

**Affiliations:** State Grid Hebei Electric Power Research Institute, Shijiazhuang, China

## Abstract

The forecast error characteristic analysis of short-term photovoltaic power generation can provide a reliable reference for power system optimal dispatching. In this paper, the total in-day error level was stratified by fuzzy C-means algorithm. Then the historical PV output data based on the numerical characteristics of point prediction output were classified. A General Gauss Mixed Model was proposed to fit the forecast error distribution of various photovoltaic output forecast error distribution. The impact of meteorological factors together with numerical characteristics on the forecast error was taken into full consideration in this analysis method. The predicted point output with high volatility can be accurately captured, and the reliable confidence interval is given. The proposed method is independent of the point prediction algorithm and has strong applicability. The General Gauss Mixed Model can meet the peak diversity, bias, and multimodal properties of the error distribution, and the fitting effect is superior to the normal distribution, the Laplace distribution, and the *t* Location-Scale distribution model. The error model has a flexible shape, a concise expression, and high practical value for engineering.

## 1. Introduction

Facing the double pressure of energy crisis and environmental pollution, people pay more and more attention to the new energy generation technology with clean and environmental protection characteristics. Compared with wind power, photovoltaic power generation requires less geographical environment and is more suitable for multiregional promotion and application. However, PV power generation is highly random and intermittent, and large-scale grid connection affects the stability and economy of the system [1]. The accuracy of photovoltaic power prediction has a direct impact on its consumption. Domestic and foreign scholars have conducted relevant studies, and the existing prediction models are divided into two categories: first, direct prediction algorithms such as regression models [2–4], gray prediction models [5–7], neural network models [8–11], and probabilistic models [12] are used; second, indirect prediction algorithms such as electronic component models [13], simple physical models [14, 15], and complex physical methods [16, 17] are used. The use of different prediction algorithms can have different degrees of prediction errors.

There are only a few literatures on the forecast error of PV power generation at home and abroad, and the description of the prediction error of PV output in some literature is based on the assumption that it obeys normal distribution. The PV output uncertainty needs to be considered when studying the optimal scheduling of power systems, and most of the literature uses the actual output value in the form of the sum of the predicted output and the forecast error. Literature [18] shows that a 10% forecast error produces deviated power exceeding 15% of the rated power value, while a 15% forecast error produces deviated power exceeding 25% of the rated power value, and the forecast error directly affects the safe and stable operation of the system. Based on the assumption that the forecast error obeys normal distribution, the results obtained in [19–21] are different from the actual statistical results. The research in [22] shows that weather factors have great influence on the forecast error, and the forecast error of solar volts in sunny days is close to normal distribution. The feasibility of using *t* Location-Scale model to describe the forecast error of PV output is proposed and verified in [23]. The statistical results show that the PV output forecast error distribution has multiple peaks, while the existing research using single distribution model is weak in describing the multipeaks. Therefore, [24–26] propose to model the forecast error by Gaussian mixture model (GMM), but the value range of GMM is from negative infinity to positive infinity, which is obviously not applicable for the description of the actual PV output forecast error directly. Literature [27] trains artificial neural networks with a large number of samples to build a forecast error model for photovoltaic power generation, which can avoid the deviation of prediction accuracy caused by model setting and parameter estimation. Literature [28] introduces regularized penalty function and error function to construct the objective function of PV prediction model; the Pearson correlation coefficient between PV power generation and each feature is analyzed, and the abnormal data of the features are also preprocessed. The above studies all focus on the optimization of the model. Because of the random characteristics of meteorological factors such as solar irradiation, temperature, and wind speed, the forecast error of photovoltaic output does not have a certain distribution characteristic, and it is difficult for the established forecast error model to achieve ideal accuracy. The distribution characteristics of PV output forecast error under different meteorological conditions and numerical characteristics cannot be ignored, so it is necessary to cluster the forecast error according to the conditions. At present, there are few researches in this field, so a flexible distribution model is needed, which can meet the requirements of skewness and peak diversity of PV output forecast error.

In this paper, the effects of meteorological and numerical characteristics on the real-time power forecast error of photovoltaic power generation are studied. Based on the corresponding meteorological data, the historical error samples are clustered into three categories by fuzzy C-means clustering, and the error areas are divided into two categories according to the error size. In order to describe the forecast error distribution more accurately, a general Gaussian mixture model based on the traditional Gaussian distribution is proposed. Compared with the traditional Gaussian model, this model can describe the error distribution of different kurtosis and shape more accurately.

In addition, this method is universal and is not affected by photovoltaic power prediction algorithm and the geographical location of photovoltaic power stations.

## 2. Cluster Analysis of Photovoltaic Output Forecast Error

Short-term forecast error of photovoltaic output is mainly affected by weather and numerical characteristics of prediction points. Among the factors representing weather, weather type, temperature, temperature difference, and wind speed are selected as indicators to analyze the correlation with photovoltaic forecast error. Therefore, firstly, the PV intraday forecast error samples are clustered into three categories according to the weather characteristics, and then the error samples obtained by classification are used as training samples to discriminate the subsequent errors. After determining the classification, the forecast error is divided into large error and small error according to its numerical characteristics. Finally, Gaussian mixture distribution is used for statistical fitting within the class, and a reliable confidence interval is provided for predicting the PV error distribution according to the fitting information.

To determine the confidence interval of photovoltaic error distribution, the steps are shown in Figure 1:

1. According to meteorological factors, the historical data of photovoltaic power generation forecast error are clustered into three categories
2. Taking amplitude and step size as indexes, the error data in cluster are divided into large error and small error
3. The error database will be established according to the error samples clustered by meteorological factors, which is convenient to provide the error interval meeting the error requirements

## 3. Influencing Factors of Photovoltaic Power Forecast Error

Photovoltaic panels absorb solar energy and generate electricity based on Volta effect. Its power generation is affected by meteorological factors, especially illumination and temperature [29]. Literature [30] proposes a photovoltaic power prediction method based on clear coefficient and multilevel similarity matching. In addition, the statistical results show that the forecast error of photovoltaic power generation is directly related to the amplitude and climbing of predicted output. Therefore, this paper studies the factors that affect the error distribution of PV power prediction from two angles of meteorological and numerical factors, which provides important reference information for error discrimination clustering and obtaining reliable confidence intervals.

### 3.1. Analysis of the Influence of Meteorological Factors on Forecast Error

To study the influence of meteorology on forecast error, we should first index meteorological factors concretely. In order to accurately scale meteorological factors, four factors are selected to express: weather type, intraday difference between maximum and minimum temperature, maximum temperature, and wind speed. After that, the influence of these four factors on forecast error is studied, which also provides variables for later error discriminant analysis.

The British statistician R. A. Fister put forward the variance analysis method in the 1920s. [31]. The variance analysis method can determine the factors that have the main effect on the target object from many factors. It determines the influence of research elements on the target object by analyzing the contribution of different elements to the overall target. The specific operation process is to analyze the differences between different groups and within groups. The specific discrimination process is as follows:

(1) $$\begin{array}{c} \left\{\begin{array}{c} \text{MSb}=\frac{\text{SSb}}{\text{dfb}},\\ \text{MSw}=\frac{\text{dfb}}{\text{dfw}}, \end{array}\right. \end{array}$$

where SSb represents the intergroup differences; SSW represents intragroup differences; dfb and dfw are the degrees of freedom between groups and within groups, respectively. Whether the experimental factors have obvious influence on the research object is judged by the ratio of MSb/MSw and the *F* distribution composed of MSb/MSw. The probability *P* value of F value greater than a specific value under the test hypothesis can be obtained by consulting the F boundary value table. Select 0.05 as the test critical value. When *P* < 0.05, it is considered that the test factors have significant differences on the research objects; otherwise, it is considered that there is no obvious influence. When studying the influence of weather factors on the forecast error of photovoltaic power generation, the selected test factors and levels are shown in Table 1.

The influence of meteorological factors on PV forecast error is analyzed. Firstly, the meteorological factors are indexed as weather type *A*, intraday temperature difference *B*, intraday maximum temperature *C*, and wind speed grade *D*. Photovoltaic forecast error is quantified by sum of squares of errors (DSSE), and weather types are quantified by sunny degree assignment [1–3]. Taking PV in Brussels area in 2016 as an example, the results of the analysis of variance are shown in Table 2.

In Table 2, the main effect of four variables and the interaction effect between two variables are selected as factors, and the sum of squares of variance, degree of freedom, mean square, observed value of *F* distribution, and test *P* value are used as indexes for analysis. As can be seen from Table 2, the *P* values of principal factor *B*, principal factor *C*, and interactive factor *B*^∗^*C* are less than 0.05. That is to say, at the significant level of 0.05, the effects of principal factor B, principal factor *C*, and interactive factor *B*^∗^*C* are significant. At the significant level of 0.05, other factors are not significant. From the results, we can see that, among the single factors selected in the early stage, factor *D* has the least significant influence on the error. In order to remove its influence on other factors and extract the components more accurately, factor *D* is removed and then does variance analysis again. The results are shown in Table 3.

As can be seen from Table 3, after removing the influence of factor *D*, the influence of factors *A*, *B*, and *C* is more significant. At a significant level of 0.05, weather type, intraday temperature difference, maximum temperature, and the interaction between intraday temperature difference and maximum temperature have the most significant influence on the total forecast error level.

### 3.2. Analysis of the Influence of Numerical Characteristics of Photovoltaic Output on Forecast Error

Photovoltaic panels usually run in the maximum power tracking state. When external factors such as illumination and temperature change, the controller controls the operating point of PV array to change, so the forecast error of photovoltaic output is related to the performance of the controller. The prediction power amplitude is selected as factor *E*, and the adjacent prediction output difference is factor *G*, and the influence of the two factors on the short-term photovoltaic output forecast error is analyzed. The rated capacity of two factors is taken as the reference value to make the standard output, and the specific level values are shown in Table 4.

Based on the photovoltaic power generation data of Brussels region in Belgium in 2016, the output amplitude and climbing power are used as indexes for principal component analysis. The results are shown in Table 5.

At a significant level of 0.05, all factors in Table 5 passed the test. Therefore, it can be seen that both the amplitude of photovoltaic output and climbing power have a significant impact on the forecast error.

### 3.3. Cluster Analysis of Influencing Factors of Photovoltaic Forecast Error

From the above analysis, it can be seen that there are many factors affecting photovoltaic forecast error. In order to facilitate the subsequent study of forecast error, it is necessary to reduce the variable dimension. In this paper, the fuzzy C-means clustering method is used to cluster the historical data DSSE, and the meteorological data are classified according to the clustering results, which can be used to discriminate and analyze the meteorological types of the forecast days and estimate the total forecast error level of the day.

Fuzzy C-mean clustering method is used in cases where there are no clear boundaries between the classified objects. Therefore, fuzzy C-means clustering method is used to combine the meteorological factors obtained above into three categories, namely, Class I, Class II, and Class III. Taking the total error level of photovoltaic prediction DSSE as the error index, the observation matrix is listed in days:

(2) $$\begin{array}{c} X=\left(\begin{array}{c} x_{1}\\ x_{2}\\ \vdots \\ x_{n} \end{array}\right)=\left(\begin{array}{ccc} x_{11} & \ldots & x_{1p}\\ \vdots & \ddots & \vdots \\ x_{n1} & \cdots & x_{np} \end{array}\right), \end{array}$$

where each row of *X* is a sample of one day and each column has *p* observations within one day; i.e., *X* is a matrix consisting of observations of *p* variables over *n* days; *X*_*np*_ represents the observed value of the *p*-th variable on the *n*-th day; *n* samples are divided into *c* classes (2 ≤ *c* ≤ *n*) and *V*={*v*_1_, *v*_2_,…*v*_*c*_} is recorded as *c* cluster centers. Samples *x*_*k*_ are not strictly divided into a certain class but belong to a certain class by membership degree *u*_*ik*_, and 0 ≤ *u*_*k*_ ≤ 1, ∑_*i*=1_^*c*^*u*_*ik*_=1. Define the target function:

(3) $$\begin{array}{c} J\left(U,V\right)=\sum_{k=1}^{n}\sum_{i=1}^{c}u_{ik}^{m}d_{ik}^{2}, \end{array}$$

where *U*=(*u*_*ik*_)_*c*×*n*_ is the membership matrix; *d*_*ik*_=‖*x*_*k*_ − *v*_*i*_‖. *J*(*U*, *V*) represents the sum of weighted square distances from samples to cluster centers in each class. Based on fuzzy C-means clustering method, Lagrange multiplier method [32] and iterative method [31] are often used to solve the objective function to obtain the minimum values of *U* and *V*.

Fuzzy C-means clustering method is used to cluster photovoltaic short-term forecast errors. The results are shown in Figure 2, where dots represent error samples. It can be seen from the figure that all error samples are clustered into three classes, and Class I error is the smallest, Class III error is the largest, and Class II error is moderate. After getting the error clustering results, the corresponding meteorological data are also classified and archived and used as their own training samples to discriminate and analyze the weather on the forecast day.

Figure 3 shows the percentage of sunny, rainy, and snowy weather on the left side and the sample mean values of intraday temperature difference, maximum temperature, and minimum temperature on the right side, which shows the clustering of meteorological data according to DSSE value clustering date. As can be seen from the above figure, the proportion of various weather types of Class I weather and Class II weather is similar, but the temperature of Class I weather is low and the temperature difference is small. The intraday temperature and temperature difference of Class II weather and Class III weather are similar, but cloudy days account for a high proportion and sunny and rainy days account for a small proportion in Class III weather.

In order to get the weather category of the forecast day, it is necessary to train each group of meteorological data as samples. In the training process, the intraday temperature difference range is [0°C, 18°C], and the intraday maximum temperature range is [−3°C, 34°C]. Mahalanobis distance, proposed by Indian statistician P.C. Mahalanobis, is a measure of similarity between two points in multidimensional space, which can effectively calculate the similarity between two unknown sample sets. Different from Euclidean distance, Mahalanobis distance between two points is independent of the measurement unit of the original data and is not affected by dimension. It can be seen from formula (4) that Mahalanobis distance is the product of Euclidean distance and spatial covariance inverse matrix. When the covariance matrix is unit matrix, Mahalanobis distance degenerates to Euclidean distance. For the factors with obvious differences, Mahalanobis distance is used to calculate the similarity, as shown in the following formula:

(4) $$\begin{array}{c} d^{2}\left(x,y\right)={\left(x-y\right)}^{T}\overset{-1}{\sum }\left(x-y\right). \end{array}$$

### 3.4. Classification Processing of Forecast Error

The research results in Section 3.2 of this paper show that the amplitude and step size of the predicted output have a significant interaction. In Section 3.2, the mean absolute error (MAE) of the samples combined by two factors at different levels is counted. The results are shown in Figure 4, and the data values are detailed in Table 6.

The statistical situation in Figure 4 is classified and described as three cases: in case 1, the combination of *E* and *G* values is missing in the lower left corner and the lower right corner of the figure, that is, {7, 1}, {8, 1}, {8, 2}, {8, 7}, {7, 8}, {8, 8} combined samples; in case 2, the dotted box area with the highest heat in the middle of Figure 2 is a large error area *E* ∈ [3,6] and *G* ∈ [3,6]; in case 3, the area that belongs neither to the large error area nor to the missing area is annularly distributed around the large error area, which is defined as the small error area.

Based on the clustering results of meteorological data, according to the characteristics of prediction output amplitude and step size, the historical data of Class I and Class II forecast errors are further divided into small error area and large error area; Class III error itself has high uncertainty and less samples, so it is no longer classified.

## 4. Forecast Error Model of Short-Term Photovoltaic Power Generation Output

### 4.1. General Gaussian Mixture Model

The statistical distribution of PV short-term output forecast error has the characteristics of asymmetry, diverse kurtosis, and multiple peaks. The traditional probability density function of Gaussian mixture distribution is defined as formula (5), where the sum of coefficients of each Gaussian term is 1.

(5) $$\begin{array}{c} f\left(x|\theta \right)=\sum_{k=1}^{n}a_{k}\phi \left(x|\theta_{k}\right), \end{array}$$

where *a*_*k*_ is the weighting factor, *a*_*k*_ ≥ 0, ∑_*k*=1_^*n*^*a*_*k*_=1; *θ*_*k*_=(*μ*_*k*_, *σ*_*k*_^2^); *ϕ*(*x|θ*_*k*_) is Gaussian distribution function as shown in the following formula:

(6) $$\begin{array}{c} \phi \left(x|\theta_{k}\right)=\frac{1}{\sqrt{2\pi }\sigma_{k}}\exp\left(-\frac{-{\left(x-\mu_{k}\right)}^{2}}{2\sigma_{k}^{2}}\right), \end{array}$$

and its cumulative distribution function is

(7) $$\begin{array}{c} F\left(x|\theta \right)=\sum_{k=1}^{n}a_{k}\int_{-\infty }^{x}\phi \left(x|\theta_{k}\right)\text{d}t. \end{array}$$

The random variable range of Gaussian mixture distribution is (−*∞*, +*∞*), but the short-term forecast error of photovoltaic is not the same in practice. To solve this problem, a general Gaussian mixture model (GGMM) is proposed based on the traditional Gaussian mixture distribution. The definition formula of GGMM is basically the same as the traditional Gaussian mixture distribution, except that there is no strict and unique restriction on the sum of the weight coefficients of each Gaussian term. Theoretically, the proposed general Gaussian mixture model is more flexible than the traditional Gaussian mixture model, and it is more applicable to describe the short-term photovoltaic output with asymmetric and multipeak characteristics.

### 4.2. Model Parameter Estimation and Accuracy Evaluation

In this paper, the least square method is used as the main method to estimate the model parameters, and the estimated parameters are obtained by the nonlinear curve fitting function lsqcurvefit in MATLAB. Multivariate determination coefficient (*R*^2^) is also called goodness of fit, and its value determines the close degree of correlation. When *R*^2^ is closer to 1, the reference value of related equations is higher. On the contrary, the closer it is to 0, the lower the reference value. Root mean square error (RMSE), also called standard error, is very sensitive to a set of extra-large or extra-small errors in fitting, so it can well reflect the precision of fitting. The closer RMSE is to 0, the higher the fitting precision is. The calculation formula is as follows:

(8) $$\begin{array}{c} \left\{\begin{array}{c} R^{2}=1-\frac{\sum {\left(y_{i}-\hat{y_{i}}\right)}^{2}}{\sum {\left(y_{i}-\bar{y}\right)}^{2}},\\ \text{RMSE}=\sqrt{\frac{\sum {\left(y_{i}-\hat{y_{i}}\right)}^{2},}{i}} \end{array}\right. \end{array}$$

where *y*_*i*_ is the actual statistical probability density, $\hat{y_{i}}$ is the curve fitting value, $\bar{y}$ is the average value, and subscript *i* represents the *i*- the error interval.

## 5. Example Analysis

In order to verify the effectiveness and applicability of the proposed method, the historical data of PV short-term prediction in Brussels, Belgium, is used as an example to simulate in MATLAB software. Among them, the historical data from 2014 to 2016 are used as training samples to establish the forecast error model, and some data from 2017 are selected as test data to test the accuracy of the model. The data in this article comes from the official website of Elia, Belgium.

Elia official website makes the next day's output forecast at 11:00 a.m. every day and updates the next day's 24-hour (96 o'clock) output at 11:45 a.m., with a time resolution of point/15 min. The collected photovoltaic output data and meteorological data have the problems of missing data and abnormal data. For the lack of intraday meteorological data, the output data of the solar photovoltaic system will not be used. And when either the predicted data or the measured data is missing and cannot be repaired, the data will not be used.

### 5.1. Comparison of Model Accuracy

In order to verify the accuracy and superiority of the model, the PV forecast error distribution model commonly used in the existing literature is used for comparison. The detailed fitting results of each model are shown in Table 7, and the fitting results are shown in Figure 5. In the figure, Emp represents the original error statistical results, 3Gau represents the proposed third-order general Gaussian mixture distribution, Lap represents Laplace distribution, *t* represents *t* Location-Scale distribution, and Nor represents normal distribution.

It can be seen from the results in Figure 5 that when the fitting distribution presents Class I and Class II small errors with higher peak degree, the accuracy of normal distribution is the lowest, followed by Laplace and Location-Scale distribution, and the proposed general Gaussian mixture distribution has the best effect. Normal distribution is obviously not enough to track spikes. When the fitting distribution shows large errors of Class I and Class II with gentle kurtosis, the effects of the three distributions mentioned above are not comparable to those of the general Gaussian mixture distribution. The fitting effect of normal distribution is better outside the peak value, but it is lower than the empirical value at the peak value. Class III error distributes gently outside the peak value but has prominent peak value. Therefore, when fitting Class III errors, the normal distribution and Laplace distribution are obviously deficient, and *t* Location-Scale is more accurate in describing the peak but obviously distorted in the nonpeak areas. The proposed general Gaussian mixture distribution has obvious advantages in describing the whole distribution. The proposed general Gaussian mixture distribution model can flexibly change the weight coefficient of each Gaussian term, so it can take into account the requirements of waist flexibility and peak value of the distribution curve and has obvious advantages in describing the short-term photovoltaic power generation output forecast error distribution.

### 5.2. Applicability Analysis of Model

In order to see whether the generalized Gaussian mixture distribution model can perform well in different meteorological environments, the historical data of different weather type days in high temperature season: July 4th (sunny day), July 8th (cloudy day), July 17th (light rain), and July 20th (thunderstorm to heavy rain) in 2017, are selected to test the applicability of the model. Using the cluster analysis method in Section 3.3, sunny days are classified as Class I generalized weather, and cloudy, light rain and thunderstorm to heavy rain are classified as Class II generalized weather. The data are counted once every 15 minutes, and the time series points with intervals of (10, 90) are selected for analysis. The model test results are shown in Figure 6.

Figure 6 shows the predicted values, measured values, and confidence interval bands of errors of photovoltaic power generation in four different weather conditions. It can be seen from the figure that the error band width of the same confidence level is different in different weather, and the error band is the narrowest in sunny days, and the worse the weather, the wider the error band. This shows that the forecast error of photovoltaic power generation is small in sunny days, and the probability of increasing the forecast error of photovoltaic power generation is greater with the deterioration of weather, which is consistent with the actual situation. In Class II and Class I weather, the difference between measured and predicted values is mainly concentrated at the peak value, while the measured curve at the waist is in good agreement with the predicted curve. This is because the peak belongs to the large error area, and the waist and bottom output belong to the small error area. Even so, the measured output at the peak is within the confidence interval of 95% of the predicted power.

In order to test the applicability of the model in low temperature season, the predicted, measured, and meteorological data of November 13, 14, 15, 16, 18, and 19, 2017 are selected in Figure 7 to test the applicability of the model to ambient temperature.

The forecast days selected in Figure 7 belong to Class I generalized weather. Similar to the test results in Figure 6, the measured values at the peak value deviate from the predicted values to a higher degree than those at the waist and bottom, but the measured values are all within the confidence interval of 95%, which shows that the model is very sensitive to the output value with large fluctuation.

To sum up, under different weather types, ambient temperatures, predicted output amplitude, and step size, the proposed general Gaussian mixture model can accurately describe the distribution of short-term PV power output forecast error, and the model has strong applicability. In addition, according to the weather conditions on the forecast day, the model can give the error bands under different confidence levels of PV short-term forecast power in advance.

## 6. Conclusion

Accurate description of wind and solar output uncertainty is the basis of establishing stochastic optimal dispatching model of power system with wind and solar power sources. In order to describe the short-term forecast error of photovoltaic power generation relatively accurately, a short-term forecast error model of photovoltaic power generation output considering meteorological factors and numerical characteristics is established in this paper, and a general Gaussian mixture model is proposed to describe the short-term forecast error of photovoltaic power generation. The model considers the influence of different meteorological conditions on the forecast error and combines numerical characteristics for analysis. Finally, taking the photovoltaic power generation system in Brussels area as an example, the effectiveness of this method is verified, and the main conclusions are as follows:

1. The short-term PV power forecast error is affected by three weather factors: weather type, temperature difference, and maximum temperature, and is also related to the output amplitude and climbing power at the predicted time
2. The general Gaussian mixture model proposed in this paper can flexibly change the weight coefficient of each Gaussian probability density, so that it can take into account the requirements of waist flexibility and peak value of distribution curve at the same time, and has obvious advantages in describing the forecast error distribution of short-term photovoltaic power generation output

In this paper, the analysis of the problem is limited by the acquisition of meteorological data. If more detailed and accurate meteorological data are obtained in the future, we can further analyze the influence of meteorological factors on the forecast error at every moment in the day and establish a more comprehensive error model in order to narrow the confidence interval and obtain more accurate results.

## Figures and Tables

**Figure 1:** Schematic diagram of the research method of photovoltaic output forecast error distribution.

**Figure 2:** Fuzzy C-means clustering results.

**Figure 3:** Clustering results of meteorological data.

**Figure 4:** MAE statistical chart of samples at each level of *E* and *G* factors.

**Figure 5:** Comparison chart of distribution fitting of five groups of errors.

**Figure 6:** The predicted value, measured value, and GGMM confidence interval under different weather in July.

**Figure 7:** The predicted value, measured value, and GGMM confidence interval under different weather in November.

**Table 1:** List of factors and levels.

Level	Factor			
	*A* (weather)	*B* (temperature difference (°C))	*C* (*T*_max_ (°C))	*D* (wind speed grade)
1	Sunny day	1∼5	-1∼10	1∼2
2	Cloudy	6∼10	11∼20	3∼4
3	Rainy day	11∼15	21∼32	5∼6

**Table 2:** Factors and test parameter values.

Source	Sum sq.	d.f.	Mean sq.	*F*	*P*
*A*	0.324	2	0.1594	1.29	0.2762
*B*	1.301	2	0.6488	5.26	0.0051
*C*	2.529	2	1.2646	10.27	≤0.0001
*D*	0.100	2	0.0501	0.41	0.6663
*A* ^∗^ *B*	0.270	4	0.0676	0.55	0.7011
*A* ^∗^ *C*	0.554	4	0.1384	1.12	0.3453
*B* ^∗^ *C*	2.909	4	0.7273	5.9	0.0001
Error	41.141	334	0.1232		
Total	51.560	354			

**Table 3:** Processed factors and processed test parameter values.

Source	Sum sq.	d.f.	Mean sq.	*F*	*P*
*A*	1.133	2	0.5650	4.62	0.0117
*B*	1.612	2	0.7983	6.57	0.0019
*C*	2.607	2	1.3001	10.77	≤0.0001
*A* ^∗^ *C*	0.655	4	0.1664	1.36	0.2886
*B* ^∗^ *C*	3.027	4	0.7374	6.16	0.0001
Error	43.225	340	0.1225		
Total	52.137	354			

**Table 4:** List of factors and levels.

Level	Factor	
	*E* (day-ahead forecast output)	*G* (step length)
1	0∼0.105	−0.06∼−0.045
2	0.105∼0.21	−0.045∼−0.03
3	0.21∼0.315	−0.03∼−0.015
4	0.315∼0.42	−0.015∼−0.003
5	0.42∼0.525	−0.003∼0.009
6	0.525∼0.63	0.009∼0.021
7	0.63∼0.735	0.021∼0.033
8	0.735∼0.84	0.033∼0.045

**Table 5:** Factors and test parameter values.

Source	Sum sq.	d.f.	Mean sq.	*F*	*P*
*E*	0.309	5	0.0539	9.36	≤0.0001
*G*	0.312	3	0.1801	15.69	≤0.0001
*E* ^∗^ *G*	1.567	43	0.0361	6.01	≤0.0001
Error	306.495	50982	0.0060		
Total	318.504	51039			

**Table 6:** The MAE statistics table of the samples of *E* and *G* factors at each level.

*E*	*G*							
	1	2	3	4	5	6	7	8
1	0.061	0.019	0.013	0.013	0.013	0.013	0.013	0.032
2	0.061	0.032	0.048	0.061	0.061	0.061	0.032	0.032
3	0.032	0.061	0.072	0.092	0.092	0.084	0.061	0.032
4	0.019	0.084	0.092	0.101	0.115	0.092	0.072	0.032
6	0.072	0.061	0.101	0.101	0.101	0.092	0.061	0.072
6	8	0.061	0.084	0.101	0.101	0.072	0.048	0.061
7	0	0.061	0.048	0.061	0.061	0.048	0.019	0
8	0	0	0.048	0.048	0.048	0.032	0	0

**Table 7:** Accuracy evaluation of different models.

	Model	*R* ^2^	RMSE
Class I small error	3GGMM	0.9856	0.0756
	Laplace	0.9326	0.8993
	*t*-distribution	0.9795	0.6865
	Normal distribution	0.8003	1.8454

Class II small error	3GGMM	0.9991	0.1027
	Laplace	0.5173	1.9803
	*t*-distribution	0.9675	0.4952
	Normal distribution	0.7264	1.5314

Class III small error	3GGMM	0.9023	0.3785
	Laplace	0.4802	0.8695
	*t*-distribution	0.7203	0.6263
	Normal distribution	0.3254	0.9886

Class I large error	3GGMM	0.9995	0.1132
	Laplace	0.9348	0.4165
	*t*-distribution	0.9951	0.1403
	Normal distribution	0.9951	0.1406

Class II large error	3GGMM	0.9601	0.1385
	Laplace	0.7784	0.4625
	*t*-distribution	0.8728	0.3098
	Normal distribution	0.8756	0.3178

## Data Availability

The data used to support the findings of this study are included within the article.

## References

[1] Wang H., Ge L., Li H., Chi F. (2017). A review on characteristic analysis and prediction method of distributed PV. *Electric Power Construction*.

[2] Wang J., Wang W., Chen H. (2019). Prediction of photovoltaic power generation based on regression-Markov chain. *Electrical Measurement and Instrumentation*.

[3] Wang Z., He L., Cheng X., He J. Method for short-term photovoltaic generation power prediction base on weather patterns.

[4] Bacher P., Madsen H., Nielsen H. (2009). Online short-term solar power forecasting. *Solar Energy*.

[5] Zhong Z., Yang C., Cao W., Yan C. (2017). Short-term photovoltaic power generation forecasting based on multivariable grey theory model with parameter optimization. *Mathematical Problems in Engineering*.

[6] Li Y., Zhang J., Xiao J., Tan Y. Short-term prediction of the output power of PV system based on improved grey prediction model.

[7] Tong C., Peng S., Xue Y. (2015). Photovoltaic power prediction based on GM-RBF neural network. *Electronic Design Engineering*.

[8] Chen Z., Yang Z., Peng Q. Study of photovoltaic short-term output predicting based on optimal algorithm.

[9] Kardakos E. G., Alexiadis M. C., Vagropoulos S. I., Simogolu C. K., Bikas P. N., Bakirzi A. G. Application of time series and artificial neural network models in short-term forecasting of PV power generation.

[10] Tang P., Chen D., Hou Y. (2016). Entropy method combined with extreme learning machine method for the short-term photovoltaic power generation forecasting. *Chaos, Solitons & Fractals*.

[11] Yang Y., Dong L. Short-term PV generation system direct power prediction model on wavelet neural network and weather type clustering.

[12] Dong L., Zhou W., Zhang P., Liu G., Li W. (2013). Short-term photovoltaic output forecast based on dynamic Bayesian network theory. *Proceedings of the CSEE*.

[13] Bae K. Y., Han S. J., Dan K. S. (2017). Hourly solar irradiance prediction based on support vector machine and its error analysis. *IEEE Transactions on Power Systems*.

[14] Yang X., Liu H., Zhang B., Xiao Y. (2014). Similar day selection based on combined weight and photovoltaic power output forecasting. *Electric Power Automation Equipment*.

[15] Zhao S., Wang M., Hu Y., Liu C. (2015). Research on the prediction of PV output based on uncertainty theory. *Transactions of China Electrotechnical Society*.

[16] Sun Y., Wang F., Zhen Z. Research on short-term module temperature prediction model based on BP neural network for photovoltaic power forecasting.

[17] Marquez R., Coimbra C. F. M. (2011). Forecasting of global and direct solar irradiance using stochastic learning methods, ground experiments and the NWS database. *Solar Energy*.

[18] Zhao B., Xue M., Chen R., Lin S. (2014). An economic dispatch model for microgrid with high renewable energy resource penetration considering forecast errors. *Automation of Electric Power Systems*.

[19] Lin S., Han M., Zhao G., Niu G. (2013). Capacity allocation of energy storage in distributed photovoltaic power system based on stochastic prediction error. *Proceedings of the CSEE*.

[20] Jiang X., Chen H., Hu X., Xiang T. (2014). A prediction error uncertainty based day-ahead unit commitment of large-scale intermittent power generation. *Power System Technology*.

[21] Li P., Zang C., Li H. (2015). Energy stochastic optimization scheduling for micro-grid based on photovoltaic forecasting. *Transducer and Microsystem Technologies*.

[22] Zhao W., Zhang N., Kang C., Wang Y., Li P., Ma S. (2015). A method of probabilistic distribution estimation of conditional forecast error for photovoltaic power generation. *Automation of Electric Power Systems*.

[23] Chen Y. (2016). Short-term photovoltaic power prediction based on typical climate types and stochastic prediction error[J]. *Electric power*.

[24] Yang M., Zhang Q. (2018). The research of ultra shortterm wind power prediction error distribution based on nonparametric estimation. *Journal of Northeast Electric Power University*.

[25] Huang Y., Cao C., Gu H. (2018). Short-term photovoltaic power generation forecasting scheme based on IKFCM and multi-mode social spider optimization SVR. *Power System Protection and Control*.

[26] Fan A., Gao S., Fang J. (2018). A PV power time series generating method considering correlation characteristics based on multi Markov chain Monte Carlo method. *Electric Power Engineering Technology*.

[27] Zhao S., Li Z. (2018). Day-ahead scheduling of multi-energy power system considering renewable energy uncertain output. *Journal of North China Electric Power University*.

[28] Peng S., Zheng G., Huang S., Lin B., Hu Z. (2020). Short-term photovoltaic power generation prediction based on XGBoost algorithm with multiple features. *Electrical Measurement and Instrument*.

[29] Lu J., Zhai H., Chun L., Wang X. (2010). Research on statistical method of photovoltaic power generation prediction. *East China Electric Power*.

[30] Wang Z., Han M., Hu H., Yao C. (2019). Research on photovoltaic power prediction method based on sunny coefficient and multi-level matching. *Electrical Measurement and Instrument*.

[31] Xie Z. (2010). *Analysis and Application of Statistics by MATLAB: Based on 40 cases*.

[32] Geng B., Gao Z., Bai H., He W., Dong W., Zhao Y. (2017). PV generation forecasting combined with similar days and GA-BP neural network. *Proceedings of the CSU-EPSA*.

